This article has been retracted.

# Ultrasound Image-Guided Nerve Block Combined with General Anesthesia under an Artificial Intelligence Algorithm on Patients Undergoing Radical Gastrectomy for Gastric Cancer during and after Operation

**DOI:** 10.1155/2022/6914157

**Published:** 2022-01-19

**Authors:** Wanqiu Fan, Liuyingzi Yang, Jing Li, Biqian Dong

**Affiliations:** ^1^Department of Anesthesiology, Affiliated Hospital of North Sichuan Medical College, Nanchong, 637000 Sichuan, China; ^2^Maternal and Child Health Hospital of Shifang, Deyang, 618400 Sichuan, China; ^3^Department of Anesthesiology, People's Hospital of Yilong County, Nanchong, 636000 Sichuan, China

## Abstract

This study was aimed at investigating the location of gastric cancer by using a gastroscope image based on an artificial intelligence algorithm for gastric cancer and the effect of ultrasonic-guided nerve block combined with general anesthesia on patients undergoing gastric cancer surgery. A total of 160 patients who were undergoing gastric cancer surgery from March 2019 to March 2021 were collected as the research objects, and the convolutional neural network (CNN) algorithm was used to segment the gastroscope image of gastric cancer. The patients were randomly divided into a simple general anesthesia group of 80 cases and a transversus abdominis plane block combined with rectus abdominis sheath block combined with the general anesthesia group of 80 cases. Then, compare the systolic blood pressure (SBP), diastolic blood pressure (DBP), and heart rate (HR) at the four time points T_0_, T_1_, T_2_, and T_3_. The times of analgesic drug use within 48 hours after operation and postoperative adverse reactions were recorded. The visual analog scale (VAS) scores were also recorded at 4 h, 12 h, 24 h, and 48 h. The results show that the image quality after segmentation is good: the accuracy of tumor location is 75.67%, which is similar to that of professional endoscopists. Compared with the general anesthesia group, the transversus abdominis plane block combined with the rectus sheath block combined with the general anesthesia group had fewer anesthetics, and the difference was statistically significant (*P* < 0.05). Compared with the general anesthesia group, SBP, DBP, and HR were significantly reduced at T_1_, T_2_, and T_3_ in the transverse abdominis plane block combined with rectus sheath block and general anesthesia group (*P* < 0.05). Compared with the simple general anesthesia group, the VAS scores of the transversus abdominis plane block combined with rectus sheath block combined with the general anesthesia group decreased at 4 h, 12 h, and 24 h after surgery, and the difference was statistically significant (*P* < 0.05). The number of analgesics used in transversus abdominis plane block combined with the rectus sheath block combined with the general anesthesia group within 48 hours after operation was significantly less than that in the general anesthesia group, and the difference was statistically significant (*P* < 0.05). The average incidence of adverse reactions in the nerve block combined with the general anesthesia group was 2.5%, which was lower than the average incidence of 3.75% in the general anesthesia group. In summary, the CNN algorithm can accurately segment the lesions in the ultrasonic images of gastric cancer, which was convenient for doctors to make a more accurate judgment on the lesions, and provided a basis for the preoperative examination of radical gastrectomy for gastric cancer. Ultrasonic-guided nerve block combined with general anesthesia can effectively improve the analgesic effect of radical gastrectomy for gastric cancer, reduced intraoperative and postoperative adverse reactions and analgesic drug dosage, and had a good effect on postoperative recovery of patients. The combined application of these two methods can further improve the precision treatment of gastric cancer patients and accelerate postoperative recovery.

## 1. Introduction

Gastric cancer is one of the most common malignant tumors in the world. It has become one of the world health problems concerned by the world because of its high incidence and poor prognosis effect, which pose a serious threat to human life, health, and quality of life [1]. At present, the treatment of gastric cancer is mainly comprehensive treatment measures of radical surgery combined with drugs and other means [2]. Laparoscopic radical surgery is the standard surgical method for radical gastrectomy of gastric cancer. Its advantages are little trauma to patients, light surgical pain, and quick recovery after surgery [3]. Laparoscopic radical gastrectomy for gastric cancer is carried out in the whole surgical process under laparoscopy, which removes the primary gastric lesions, infiltrating tissues involved in the primary gastric lesions, and lymph nodes involved around the stomach at one time. All gastric lesions affected by tumors can be completely removed by a single operation to achieve a cure effect [4]. Although laparoscopic radical gastrectomy is an effective treatment for gastric cancer, the immune function of patients is impaired due to trauma, pain, and other reasons during the operation. The postoperative pain of patients is aggravated, and the possibility of gastric cancer recurrence is greatly increased, which is extremely harmful to the postoperative prognosis of patients [5].

The postoperative trauma of radical gastrectomy for gastric cancer is mainly severe pain. During surgery, the number of T lymphocytes and natural killer cells will be reduced, and their activity will be weakened, resulting in disruption of the dynamic balance of regulatory T lymphocytes, helper T lymphocytes, and cytotoxic T lymphocytes in the body. These cells have a great influence on the immune system and the degree of surgical trauma [6]. The original analgesic methods include oral opioid analgesics, intramuscular injection of dolantin and other analgesic injection, and local administration. A single analgesic method often produces an obvious and rapid analgesic effect on severe pain after radical gastrectomy [7]. In recent years, ultrasound-guided nerve block and other multimodal analgesia, such as transversus abdominis plane block combined with rectus abdominis sheath block, have gradually been used clinically. The main principle is to block the signal transduction pathway which can maximize the control of postoperative pain in patients [8].

With the rapid development of computer technology and the update of hardware equipment, the artificial intelligence algorithm has been gradually applied in the analysis and diagnosis of specific diseases in medical imaging based on the characteristics of the artificial intelligence algorithm, which can reach the diagnosis level of lesions with professional imaging physicians or even more accurate. Machine learning is one of the ways to realize artificial intelligence algorithms [9]. It includes a variety of algorithms, such as the Bayesian algorithm, linear classifier, cluster analysis algorithm, and convolutional neural network (CNN) algorithm [10]. Pham et al. [11] used three-dimensional supervoxels in artificial intelligence algorithms to conduct in-depth analysis of MRI images in databases with sample sizes of 11 and 30 and found that the similarity coefficients were 0.84 and 0.89. It shows that the artificial intelligence algorithm has high accuracy in segmentation of MRI image lesions, and it has great clinical application value. A type of CNN algorithm in artificial intelligence algorithms has attracted more attention in medical research. It is a deep learning model evolved from biological concepts, which can classify, recognize, and segment images [12]. Therefore, this study analyzed the location of gastric cancer by using a gastroscope image based on the artificial intelligence algorithm for gastric cancer and the effect of ultrasonic-guided nerve block combined with general anesthesia on patients undergoing radical gastritis, hoping to provide a new method of anesthesia for patients undergoing radical gastric cancer surgery. In addition, artificial intelligence algorithms are used to assist clinical imaging in the diagnosis of gastric cancer, which provides a reference.

## 2. Methods

### 2.1. Research Objects

A total of 160 patients who were undergoing gastric cancer surgery from March 2019 to March 2021 were collected as the research objects. They were randomly divided into a general anesthesia group of 80 cases and a transverse abdominis plane block combined with rectus abdominis sheath block and general anesthesia group of 80 cases (nerve block general anesthesia group). There were 99 male patients and 61 female patients. The age was 36~68 years, with a mean age of 52.3 ± 3.64 years.

Inclusion criteria were as follows: (i) patients were diagnosed with primary gastric cancer by professional doctors; (ii) preoperative abdominal and chest CT examination of all patients showed no other metastasis; (iii) all clinical information of patients was complete; (iv) the patient had no other serious complications, including organ function impairment of the heart, liver, lung, and kidney; and (v) no surgical contraindications were found.

Exclusion criteria were as follows: (i) the patient had other gastric complications, such as gastrointestinal dysfunction; (ii) patients had autoimmune diseases, such as autoimmune hemolytic anemia; (iii) patients had acute or chronic infectious diseases; (iv) patients had mental or consciousness disorders and poor compliance; and (v) the patient had a recent history of surgical treatment and special medication.

All patients in this study and their authorized family members had signed informed consent, and the study had been approved by the Medical Ethics Committee of the Affiliated Hospital of North Sichuan Medical College.

### 2.2. Ultrasound Gastroscopy

In this study, a Mindray ultrasonic diagnostic instrument was used in this study. The patients were fasted for six hours before the test. Dyclonine hydrochloride mucilage is taken before examination. Assist the patient to take the left decubitus position with calm breath. The gastroscopy probe was passed through the mouth and the esophagus into the stomach; select the best image to display the lesion location of the patient.

### 2.3. Segmentation of the Ultrasound Image Based on CNN

Classic CNN consists of an input layer, convolution layer, pooling layer, full connection layer, and output layer. Its structure is shown in Figure 1. CNN starts from the input to the output. Each layer is connected with each other through its own mathematical operation, and then, information is transferred to the next layer through the connection. Several convolution operations and pooling operations decode, analyze, and cluster the characteristic signals of the input original image data and finally map them to specific spatial layers. The final data information is classified and output by the full connection layer according to the target characteristics.

The operation between the convolutional layer and the pooling layer is mainly realized through a series of mathematical function operations. The convolutional layer is also called the feature extraction layer, which is used to extract the feature region of interest from the input raw data. Each convolutional layer has its corresponding convolution kernel. If the convolution kernel is different, the extracted features will be different. The more convolution kernels in each layer, the more features can be extracted in the convolution layer. The convolution operation is mainly realized by the convolution operation. The mathematical equation of convolution operation is shown in

(1) $$\begin{array}{c} y\left(t\right)=\int_{-\infty }^{\infty }f\left(x-\tau \right)h\left(\tau \right)d\tau . \end{array}$$

In the process of medical image processing, if a two-dimensional image is used as input data and input to the convolutional layer, the convolution operation will become

(2) $$\begin{array}{c} y\left(x,y\right)=\int \int f\left(a,b\right)t\left(x-a,y-b\right)dadb. \end{array}$$

At present, most studies will give a convolution kernel of a prescribed size, and the complete convolution operation is

(3) $$\begin{array}{c} y\left(x,y\right)=\overset{a=A}{\underset{a=0}{\sum }}\overset{b=B}{\underset{b=0}{\sum }}f\left(a,b\right)t\left(x-a,y-b\right). \end{array}$$

Among them, *y*(*x*, *y*) represents the output result, *f*(*a*, *b*) represents the input data, and the size of the convolution kernel is *A* × *B*.

The pooling layer is used to effectively delete the remaining data while retaining the characteristic data of the upper convolution result, reduce processing parameters, and speed up the extraction speed. The pooling layer operation is divided into average extraction and maximum extraction. At present, the most researched is the maximum value extraction. The maximum pooling operation is shown in Figure 2.

### 2.4. Anesthesia Methods

All patients were monitored by heart rate, blood pressure, electrocardiogram, and SpO_2_. Intravenous induction of general anesthesia was performed by using 0.3 *μ*g/kg sufentanil, 0.15 mg/kg cisatracurium, and 2 mg/kg propofol. Then, tracheal intubation was performed three minutes later. After tracheal intubation, intraoperative anesthesia was inhaled with 2% sevoflurane and pumped with 0.1 *μ*g/kg/min remifentanil. 0.06 mg/kg cisatracurium was injected intermittently every hour to maintain anesthesia depth, 0.2 *μ*g/kg sufentanil was given at the beginning of incision closure, and all anesthesia was stopped after skin suture. General anesthesia was performed combined with nerve block which means that before induction of general anesthesia, 0.33% ropivacaine was given for transverse fascia block and rectus sheath block, 20 ml for each part. The general anesthesia plan was the same as the one above, and 0.15 mg/kg dezocine was given if the patient was in unbearable pain after surgery.

### 2.5. Evaluation Index of Image Segmentation

Accuracy was used as an index to quantitatively evaluate the results of image segmentation. Accuracy indicates the degree to which the algorithm can correctly segment the diseased area. The index is defined as follows.

(4) $$\begin{array}{c} \text{Accuracy}=\frac{\text{TP}+\text{TN}}{\text{TP}+\text{TN}+\text{FP}+\text{FN}}, \end{array}$$

where TP indicates that the segmentation result is a diseased area, which is actually also a diseased area. TN segmentation results show that it is not a lesion area, nor is it actually a lesion area. FP indicates that the segmentation result is a diseased area, which is not actually a diseased area. FN indicates that the segmentation result is not the lesion area, which is actually the lesion area.

### 2.6. Surgical Evaluation Indexes

Systolic blood pressure (SBP), diastolic blood pressure (DBP), and heart rate (HR) of patients were evaluated at preinduction of anesthesia time point (T_0_), at the beginning of the operation (T_1_), 30 min intraoperatively (T_2_), and 1 h intraoperatively (T_3_). The visual analog scale (VAS) scores were determined at 4 h, 12 h, 24 h, and 48 h after surgery. In this study, a score of 0 indicated that the patient had no pain and a score of 10 indicated that the patient had unbearable pain. Postoperative adverse reactions: dizziness, headache, nausea and vomiting, hypotension.

### 2.7. Statistical Analysis

All data in this study were analyzed by using SPSS 20.0. Measurement data were expressed in the form of mean ± standard deviation, and the *t*-test was used in the group. The chi-square test was used for counting data. When *P* < 0.05, the difference was statistically considerable.

## 3. Results

### 3.1. Basic Data of the Two Groups of Patients

There were no considerable differences in gender, age, body mass index, operation time, and blood loss during operation between 80 patients in the general anesthesia group and 80 patients in the nerve block general anesthesia group (*P* > 0.05), and the two groups were comparable subsequently.  Table 1 shows the details.

### 3.2. Image Segmentation Results of the CNN Algorithm

The gastroscopic images of gastric cancer patients were segmented, and the proposed CNN algorithm was compared with the lesion location of imaging professionals. The result is shown in Figure 3. Diagnosis and positioning statistics of professional physicians were reported by gastroscopy, the localization effect of the lesion area in the image segmented by the CNN algorithm is similar to that of the doctor's manual localization, and the lesion area is clear. It is proven that the CNN algorithm has good application value in the image localization of gastric cancer patients.

### 3.3. Comparison of Evaluation Indicators of Segmentation Results

In this study, the localization results of lesions using the CNN algorithm were evaluated by accuracy. The result is shown in Figure 4. The accuracy of imaging doctors in determining tumor location was 72.38%, while the accuracy of the CNN algorithm was 75.67%. Compared with the judgment of tumor location by professional imaging doctors, the judgment of tumor location by the CNN algorithm is similar to that by professional imaging doctors. The research proves that the CNN algorithm proposed in this paper can be used for clinical image positioning.

### 3.4. Comparison of SBP, DBP, and HR between the Two Groups of Patients at Various Time Points

The comparison results of SBP, DBP, and HR indexes of the two groups of patients at four time points are shown in Figure 5. The three indexes of the nerve block general anesthesia group of patients were lower at T_0_ than at the T_1_, T_2_, and T_3_ time points, while the general anesthesia group was higher at T_0_ than at the T_1_ time point (*P* < 0.05), and there was no statistical significance at T_2_ and T_3_. Compared with the general anesthesia group, the SBP, DBP, and HR of the nerve block general anesthesia group at the T_1_, T_2_, and T_3_ time points all decreased, and the differences were statistically significant (*P* < 0.05).

### 3.5. Postoperative General Anesthetic Use and VAS Score Results of the Two Groups of Patients

The number of analgesics used within 48 hours after surgery of the two groups and the results of the VAS score are shown in Table 2. The number of analgesics used of the general anesthesia nerve block group after radical gastrectomy was dramatically less than that of the general anesthesia group alone, and the difference was considerable (*P* < 0.05). Compared with the general anesthesia group, the VAS scores of the nerve block general anesthesia group were lower at 4 h, 12 h, and 24 h after surgery which were dramatically different (*P* < 0.05).

### 3.6. Comparison of Adverse Reactions between the Two Groups of Patients after Surgery

By comparing the incidence of adverse reactions between the two groups of patients, the postoperative clinical evaluation indexes of the two groups of patients were evaluated. The results are shown in Table 3. The average incidence of adverse reactions in the general anesthesia group after nerve block was 2.5%, which was lower than the average incidence of 3.75% in the general anesthesia group. It showed that the incidence of adverse reactions after radical gastric cancer in the general anesthesia group of nerve block was lower.

## 4. Discussion

As one of the common malignant tumors of the digestive system, gastric cancer has very high morbidity and mortality. The overall incidence of gastric cancer occupies the second place among all malignant tumors, and the mortality rate occupies the third place among all malignant tumors [13]. According to the *2018 Global Cancer Statistics Report*, there are about 18.19 million new cases of cancer worldwide and more than 9.6 million deaths due to cancer. Stomach cancer is the third leading cause of death among all cancers. In addition, the morbidity and mortality of male patients were higher than those of female patients. Due to differences in diet structure, food storage, and other factors, Asian people have a higher risk of gastric cancer compared to people from other regions [14, 15]. Korea has the highest incidence and fatality rate of stomach cancer among Asian countries. Since the symptoms of gastric cancer in the early stage are secretive and have no typical clinical manifestations, patients may only have mild gastrointestinal discomfort, which is therefore ignored by most patients [16–18]. Once the symptoms worsen, gastric cancer is in the advanced stage and the optimal treatment window has been missed. Therefore, the 5-year survival rate of gastric cancer patients is less than 30% [19].

With the continuous development of computer technology, the artificial intelligence algorithm has gradually been widely used in cancer treatment. Artificial intelligence algorithms include a supervised learning algorithm, unsupervised learning algorithm, clustering algorithm, and dimensionality reduction [20]. The classical CNN algorithm is one of the commonly used artificial intelligence algorithms. It combines modern computer technology with traditional medical imaging. On the one hand, it helps clinicians mine more detailed and accurate image information of patients' imaging data through the CNN algorithm and guides doctors to provide more personalized diagnosis and treatment plans for patients. On the other hand, the data can be stored in the computer for a long time and accumulated at a large scale, so as to realize the early prediction of certain diseases [21]. This study compared the segmentation results of gastroscopic images of gastric cancer patients by the CNN algorithm and professional doctors. The results show that the CNN algorithm has high image quality, clear image, and accurate lesion range and can accurately locate the tumor. The segmentation results were similar to those of professional doctors. The results show that the CNN algorithm has good clinical application value in tumor localization.

Currently, surgery is the most common treatment for gastric cancer. In clinical treatment, radical gastrectomy for gastric cancer is mostly carried out under laparoscopy, and the original general anesthesia requires a large number of opioid analgesics, which have obvious analgesic effect. However, postoperative patients are prone to stress reactions, such as dizziness, headache, nausea, and vomiting, which will also affect the immune function of patients, especially adverse to the prognosis of patients. Based on this, experts from the Chinese Society of Anesthesiology proposed multimode analgesia, such as ultrasound-guided nerve block combined with general anesthesia. This comprehensive analgesic method can not only effectively control patients' postoperative pain but also play a role in the related adverse reactions caused by pain [22]. The results of this study showed that, compared with the simple general anesthesia group, the ultrasound-guided transversus abdominis plane block combined with the rectus abdominis sheath block anesthesia group used significantly less anesthetics during radical gastric cancer surgery than the simple general anesthesia group. The difference was statistically significant (*P* < 0.05), and the average incidence of adverse reactions in patients was 2.5%, which was lower than the average incidence of adverse reactions in the simple general anesthesia group of 3.75%.

Studies suggested that the VAS scores within 24 h after surgery of ultrasound-guided transversus abdominis plane block combined with the rectus abdominis sheath block were reduced compared with those of the control group using general anesthesia alone [23]. The results of this study showed that the VAS scores of the ultrasound-guided transversus abdominis plane block combined with rectus sheath block anesthesia group at 4 h, 12 h, and 24 h after surgery were lower than the VAS scores at the corresponding time in the general anesthesia group (*P* < 0.05). Compared with the general anesthesia group, the transversus abdominis plane block combined with the rectus abdominis sheath block anesthesia group was at T_1_, T_2_, and T_3_. At the time point, SBP, DBP, and HR all decreased. It is suggested that the ultrasound-guided transversus abdominis plane block combined with rectus abdominis sheath block anesthesia group has a better effect on the intraoperative and postoperative improvement of gastric cancer patients than the simple general anesthesia group.

## 5. Conclusion

Through this study, it is found that the artificial intelligence algorithm can accurately segment the imaging lesions, helping doctors to provide more accurate diagnosis and treatment plans for patients. Ultrasonic-guided nerve block combined with general anesthesia can effectively improve the analgesic effect of radical gastrectomy for gastric cancer, reduce the adverse reactions and analgesic drug dosage during and after operation, and have a good helping effect on postoperative recovery of patients. The application of the above two methods can improve the precision treatment of gastric cancer surgery patients and accelerate the recovery of patients.

## Figures and Tables

**Figure 1:** The basic structure of CNN.

**Figure 2:** Principle of maximum pooling.

**Figure 3:** Results of lesion segmentation by the CNN algorithm.

**Figure 4:** Comparison of tumor positioning judgment result between imaging professional doctors and CNN algorithm (A: results given by the imaging doctor; B: results obtained by using the CNN algorithm).

**Figure 5:** The results of the two groups of patients on the three indexes of SBP, DBP, and HR: (a) the SBP results of the two groups of patients at the time points of T_0_, T_1_, T_2_, and T_3_; (b) the DBP results of the two groups of patients at T_0_, T_1_, T_2_, and T_3_; (c) the HR results of the two groups of patients at T_0_, T_1_, T_2_, and T_3_. Compared with general anesthesia at T_0_ (^A^*P* < 0.05); compared with nerve block general anesthesia at T_0_ (^C^*P* < 0.05); compared with nerve block general anesthesia (^B^*P* < 0.05).

**Table 1:** Basic data of patients in the two groups.

Group	Number	Age	Sex (*n*)		BMI (kg/m^2^)	Length of operation (h)	Bleeding volume (mL)
			Male	Female			
General anesthesia group	80	51.21 ± 2.73	51	29	22.23 ± 3.21	3.94 ± 0.41	208.19 ± 85.31
Nerve block general anesthesia	80	52.50 ± 3.62	48	32	23.67 ± 2.53	3.73 ± 0.72	210.67 ± 109.65

**Table 2:** Postoperative general anesthetic use and VAS score results of the two groups of patients.

Group	Number	Analgesic (time)	VAS score			
			4 h	12 h	24 h	48 h
General anesthesia group	80	6.14 ± 2.33	4.06 ± 0.81	4.59 ± 0.74	5.15 ± 0.77	3.05 ± 0.65
Nerve block general anesthesia group	80	3.17 ± 1.81^∗^	1.96 ± 0.68^∗^	2.11 ± 0.85^∗^	2.39 ± 0.74^∗^	2.43 ± 0.67

Compared with the general anesthesia group (^∗^*P* < 0.05).

**Table 3:** Comparison of adverse reactions between two patients.

Group	Dizziness and headache	Nausea and vomiting	Low blood pressure	Average incidence
General anesthesia group	4 (5%)	2 (2.5%)	3 (3.75%)	3.75%
Nerve block general anesthesia group	3 (3.75%)	1 (1.25%)	2 (2.5%)	2.5%

## Data Availability

The data used to support the findings of this study are available from the corresponding author upon request.

## References

[1] Poorolajal J., Moradi L., Mohammadi Y., Cheraghi Z., Gohari-Ensaf F. (2020). Risk factors for stomach cancer: a systematic review and meta-analysis. *Epidemiol Health*.

[2] Nunobe S., Kumagai K., Ida S., Ohashi M., Hiki N. (2016). Minimally invasive surgery for stomach cancer. *Japanese Journal of Clinical Oncology*.

[3] Venneman K., Huybrechts I., Gunter M. J., Vandendaele L., Herrero R., Van Herck K. (2018). The epidemiology of Helicobacter pylori infection in Europe and the impact of lifestyle on its natural evolution toward stomach cancer after infection: a systematic review. *Helicobacter*.

[4] Deng W., Jin L., Zhuo H., Vasiliou V., Zhang Y. (2021). Alcohol consumption and risk of stomach cancer: a meta-analysis. *Chemico-Biological Interactions*.

[5] Bui Q. L., Grazziotin-Soares D., Hasiniatsy R. E. (2018). Metastatic stomach cancer: clinical trials in Asia and in Occident. *Bulletin du Cancer*.

[6] Gu E., Song W., Liu A., Wang H. (2020). SCDb: an integrated database of stomach cancer. *BMC Cancer*.

[7] Peng W. J., Jia X. J., Wei B. G., Yang L. S., Yu Y., Zhang L. (2015). Stomach cancer mortality among workers exposed to asbestos: a meta-analysis. *Journal of Cancer Research and Clinical Oncology*.

[8] Morrison M. E. W., Joseph J. M., McCann S. E., Tang L., Almohanna H. M., Moysich K. B. (2020). Cruciferous vegetable consumption and stomach cancer: a case-control study. *Nutrition and Cancer*.

[9] Suh M., Wikoff D., Lipworth L. (2019). Hexavalent chromium and stomach cancer: a systematic review and meta-analysis. *Critical Reviews in Toxicology*.

[10] Soltaninejad M., Yang G., Lambrou T. (2018). Supervised learning based multimodal MRI brain tumour segmentation using texture features from supervoxels. *Computer Methods and Programs in Biomedicine*.

[11] Pham T. M., Quy P. N., Horimatsu T. (2020). Premature mortality due to stomach cancer in Japan: a nationwide analysis from 1980 to 2015. *Annals of Epidemiology*.

[12] Welling R., Beaumont J. J., Petersen S. J., Alexeeff G. V., Steinmaus C. (2015). Chromium VI and stomach cancer: a meta-analysis of the current epidemiological evidence. *Occupational and Environmental Medicine*.

[13] Zhang K., Yin J., Huang H. (2020). Expenditure and financial burden for stomach cancer diagnosis and treatment in China: a multicenter study. *Frontiers in Public Health*.

[14] Phuoc L. H., Sengngam K., Ogawa T. (2020). Fruit and vegetable intake and stomach cancer among male adults: a case-control study in northern Viet Nam. *Asian Pacific Journal of Cancer Prevention*.

[15] Hejna M., Wöll E., Tschandl P., Raderer M. (2016). Cutaneous paraneoplastic disorders in stomach cancer: collaboration between oncologically active dermatologists and clinical oncologists. *Critical Reviews in Oncology/Hematology*.

[16] Ruiz E. F., Torres-Roman J. S., Servan S. A. (2019). Trends and geographic pattern of stomach cancer mortality in Peru. *Cancer Epidemiology*.

[17] Kim J., Hyun H. J., Choi E. A., Kim Y., Bae Y. J., Kang H. T. (2020). Metformin use reduced the risk of stomach cancer in diabetic patients in Korea: an analysis of Korean NHIS-HEALS database. *Gastric Cancer*.

[18] Chernousov A. F., Khorobrykh T. V., Vychuzhanin D. V., Kharlov N. S., Nurutdinov R. (2018). Subcutaneous port systems with intraperitoneal catheter 'BBraun' in combined treatment of advanced stomach cancer. *Khirurgiya. Zhurnal im. N.I. Pirogova*.

[19] Lee J. H., Kim D. H., Jeong S. N., Choi S. H. (2018). Detection and diagnosis of dental caries using a deep learning-based convolutional neural network algorithm. *Journal of Dentistry*.

[20] Anwar S. M., Majid M., Qayyum A., Awais M., Alnowami M., Khan M. K. (2018). Medical image analysis using convolutional neural networks: a review. *Journal of Medical Systems*.

[21] Kearney V., Haaf S., Sudhyadhom A., Valdes G., Solberg T. D. (2018). An unsupervised convolutional neural network-based algorithm for deformable image registration. *Physics in Medicine and Biology*.

[22] Dahou A., Elaziz M. A., Zhou J., Xiong S. (2019). Arabic sentiment classification using convolutional neural network and differential evolution algorithm. *Computational Intelligence and Neuroscience*.

[23] Liu R., Qin H., Wang M., Li K., Zhao G. (2019). Transversus abdominis plane block with general anesthesia blunts the perioperative stress response in patients undergoing radical gastrectomy. *BMC Anesthesiology*.

